This article has been retracted.

# Effect of Adiponectin on Kidney Crystal Formation in Metabolic Syndrome Model Mice via Inhibition of Inflammation and Apoptosis

**DOI:** 10.1371/journal.pone.0061343

**Published:** 2013-04-22

**Authors:** Yasuhiro Fujii, Atsushi Okada, Takahiro Yasui, Kazuhiro Niimi, Shuzo Hamamoto, Masahito Hirose, Yasue Kubota, Keiichi Tozawa, Yutaro Hayashi, Kenjiro Kohri

**Affiliations:** Department of Nephro-urology, Nagoya City University Graduate School of Medical Sciences, Nagoya, Japan; Juntendo University School of Medicine, Japan

## Abstract

The aims of the present study were to elucidate a possible mechanism of kidney crystal formation by using a metabolic syndrome (MetS) mouse model and to assess the effectiveness of adiponectin treatment for the prevention of kidney crystals. Further, we performed genome-wide expression analyses for investigating novel genetic environmental changes. Wild-type (+/+) mice showed no kidney crystal formation, whereas ob/ob mice showed crystal depositions in their renal tubules. However, this deposition was remarkably reduced by adiponectin. Expression analysis of genes associated with MetS-related kidney crystal formation identified 259 genes that were >2.0-fold up-regulated and 243 genes that were <0.5-fold down-regulated. Gene Ontology (GO) analyses revealed that the up-regulated genes belonged to the categories of immunoreaction, inflammation, and adhesion molecules and that the down-regulated genes belonged to the categories of oxidative stress and lipid metabolism. Expression analysis of adiponectin-induced genes related to crystal prevention revealed that the numbers of up- and down-regulated genes were 154 and 190, respectively. GO analyses indicated that the up-regulated genes belonged to the categories of cellular and mitochondrial repair, whereas the down-regulated genes belonged to the categories of immune and inflammatory reactions and apoptosis. The results of this study provide compelling evidence that the mechanism of kidney crystal formation in the MetS environment involves the progression of an inflammation and immunoresponse, including oxidative stress and adhesion reactions in renal tissues. This is the first report to prove the preventive effect of adiponectin treatment for kidney crystal formation by renoprotective activities and inhibition of inflammation and apoptosis.

## Introduction

The worldwide prevalence of kidney stone formation increased in the last quarter of the 20th century [1]. A change in diet, especially an increased intake of lipid and animal protein, is believed to be a cause of this increased prevalence of kidney stones. The prevalence of obesity, hypertriglyceridemia, and hypercholesterolemia shows a high correlation with that of kidney stones [2].

The major components of kidney stones are inorganic materials, with a small percentage of organic material called stone matrix; 90% of the inorganic components are calcium salts, of which the majority is calcium oxalate (CaOx) [3], [4]. Asplin *et al.* stated that excretion values and concentrations of urinary CaOx could not be identified as risk factors [5].

In our previous studies, we detected osteopontin (OPN) as a stone matrix protein [6] and reported an increase in renal OPN expression by using a crystal formation animal model [7]. We performed microarray analysis using the crystal forming mouse kidneys, and found increased expression of inflammation-related genes such as Monocyte Chemoattractant Protein-1 (MCP-1) and decreased expression of lipid metabolism-related genes such as adiponectin (APN) [8]. We also reported renal proximal tubular cell injury and oxidative stress caused by a mitochondrial disorder in the early phase of kidney crystal formation [9]. This mechanism of kidney crystal formation is very similar to that of atherosclerosis and was the basis of our hypothesis that kidney crystal formation is a metabolic syndrome (MetS)-related disease.

Recently, kidney stone formation has been recognized as a MetS-related disease [10]–[13]. Taylor *et al.* reported a positive relation between obesity, weight gain, and the risk of kidney stones in a prospective study of 3 large cohorts [10]. Moreover, researchers have shown an epidemiological association between atherosclerosis and kidney stones. Yasui *et al.* showed a high association between aortic calcification index and kidney stones, as detected by Computed Tomography [13].

A recent study has suggested that a decrease in APN, a fat-derived hormone, is involved in MetS pathology, and that APN reverses insulin resistance associated with both lipoatrophy and obesity [14]. Matsuda *et al.* [15] reported that APN administration could prevent vascular stenosis. Yamauchi *et al.* [16] showed that leptin-deficiency reversed insulin resistance in ob/ob mice and that APN administration could prevent atherosclerosis. Moreover, APN supplementation ameliorated renal fibrosis, diabetes nephropathy, and albuminuria in ob/ob mice [17]. Taken together, APN has antiatherosclerotic, renoprotective, anti-inflammatory, and antioxidative functions, and might be an ideal preventive medicine for kidney stones.

Here, we evaluated kidney crystal formation in a MetS mouse model, ob/ob mice. Moreover, we investigated the genetic environmental changes in the kidney using genome-wide analysis to explore the possible mechanism of kidney crystal formation in the MetS environment and the amelioration by APN.

## Materials and Methods

### Animals and genotyping

B6.V-Lep^ob/ob^ (designated here as ob/ob) and B6.V-Lep^+/+^ (designated here as +/+) (Charles River Japan, Yokohama, Japan) male mice were acclimated at 23±1°C on a 12-h light/dark cycle before initiation of experiments. All experiments were conducted using 8-week-old male littermates. All animals had free access to water and standard chow (Oriental Yeast Co., Tokyo, Japan). The genotypes of the progeny from heterozygous crossings were determined with TaqMan genotyping assays using genomic DNA extracted from tail tissue by using original, designed TaqMan probe sets (Applied Biosystems, Foster City, CA, USA). This study was carried out in strict accordance with the Guide for the Care and Use of Laboratory Animals of the National Institute of Health. All experiments were approved by the Animal Care Committee of the Faculty of Medicine, Nagoya City University Graduate School of Medical Sciences (Permit Number: H19-34). All surgery was performed under sodium pentobarbital anesthesia, and all efforts were made to minimize suffering.

CaOx crystal deposition was induced in male ob/ob mice (V-Lep^ob/ob^, 8 wk of age, *n* = 12) and +/+ mice (V-Lep^+/+^, 8 wk of age, *n* = 12) by administering 50 mg/kg glyoxylate (GOx) for 6 days, as previously described [7].

### APN treatment

Mice were treated with APN (Recombinant Mouse gAdiponectin/gAcrp30, R&D Systems, Inc., Minneapolis, USA) by subcutaneous injection in the back of each mouse for 6 days at the same time of administering glyoxylate. The amount of APN administered per day was 2.5 µg/ml in a total volume of 0.2 ml of PBS with a clean 27-gauge needle.

### Serum and urine biochemistry and detection of kidney crystal formation

On days 0 and 6, kidneys were extracted, and the right unilateral kidney specimens were stored with RNAlate (Ambion, CA, USA) at −70°C until RNA preparation, and the contralateral specimens were fixed in 4% paraformaldehyde and embedded in paraffin. All mice were placed in metabolic cages on days 1 and 5. Before kidney extraction, 24-h urine samples were collected. Urinary volume, pH, calcium, phosphorus, magnesium, oxalate, and citrate were determined at each time point (SRL, Tokyo, Japan). Serum samples were collected just before kidney extraction, and calcium, phosphorus, creatinine, TG, TC, and FFA concentrations were determined at each time point (SRL, Tokyo, Japan). The amount of crystals was determined as previously described [7].

### Microarray analysis and data mining

We prepared cRNA and conducted microarray analyses at Bio Matrix Research using the Affymetrix system (Santa Clara, CA, USA). Isolated total RNA (1 mg) was converted into double-stranded cDNA by using the One-Cycle cDNA Synthesis Kit (Affymetrix), which was purified using a GeneChip Sample Cleanup Module (Affymetrix). In vitro transcription reactions were performed using a GeneChip IVT Labeling Kit, which includes T7 RNA polymerase and biotin-labeled ribonucleotides. Biotin-labeled cRNA was purified using a GeneChip Sample Cleanup Module. The cRNA concentration was calculated from light absorbance at 260 nm using a UV spectrophotometer. Next, cRNA (15 mg) was fragmented at 94°C in the presence of a fragmentation buffer (Affymetrix). The labeled cRNA was purified, fragmented, and spiked with in vitro transcription controls. Fifteen micrograms of cRNA was hybridized using the GeneChip Mouse Genome 430 2.0 Array (Affymetrix). The array was incubated for 16 h at 45°C and automatically washed and stained with the GeneChip Hybridization, Wash, and Stain Kit (Affymetrix) on an Affymetrix GeneChip Fluidics station. The probe array was scanned using a GeneChip Scanner 30007G.

The value of the transcript was calculated with the 11 values of perfect match (PM) and mismatch (MM) probes by using the GeneChip Operating Software (GCOS), in which the probabilities of the values of each transcript were indicated as “Flag” Present (p≥0 to <0.04), Marginal (p≥0.04 to <0.06), or Absent (p≥0.06 to <0.5), using one-sided Wilcoxon's signed rank test between the values of PM and MM. Analysis, normalizations, relative signal intensities, and fold changes between GOx-treated (day 6) and control samples (day 0) were calculated using GeneSpring GX 11.0 (Agilent Technologies, Loveland, Colorado, USA) data-mining software. For the extraction of kidney crystal formation-related genes, the Venn diagram function appended with the GeneSpring software was used to select genes whose expression changed by >2.0 fold and <0.5 fold. The sorted gene lists were analyzed with the GO ontology browser, one of the functions of GeneSpring GX 11.0, and the categories of biological process, cellular components, and molecular function were sorted on the basis of the annotation of listed genes. The *p* value of each category was calculated using Fisher's exact test. And we registered our data of microarray analysis data to the Gene Expression Omnibus of the *National Center for Biotechnology Information* (GEO accession number; GSE37173).

### Quantitative PCR

Total RNA was isolated from frozen sections of mouse kidney samples with an RNeasy Midi Kit (Qiagen Co., Düsseldorf, Germany) according to the manufacturer's instructions. TaqMan Gene Expression Assay (Applied Biosystems, Foster City, CA,USA), 20× assay mix of primers, and TaqMan MG probes (FAM dye labeled; Applied Biosystems) were used for quantitative RT-PCR. This assay was designed to span exon–exon junctions so as not to detect genomic DNA. Validation experiments were performed to test the efficiency of the target amplification and reference amplification. The materials used for and genes analyzed by quantitative RT-PCR with the ABI PRISM 7700 Sequence Detection System (Applied Biosystems) are listed in Table S11. The primers and probe sequences were searched against the Celera database to confirm specificity. Validation experiments were performed to test the efficiency of the target amplification and reference amplification. Beta-actin (*Actb*, Mm00456425_m1) was used as the inner control for gene expression.

### Immunohistochemical staining

Immunohistochemical staining was carried out on 4-µm-thick cross-sections. Sections were microwave treated for 15 min and blocked with 0.5% H_2_O_2_ in methanol for 30 min, washed in 0.01 M PBS, and further treated with skim milk in PBS for 1 h at room temperature. These slides were incubated overnight at 4°C with the antibodies listed in Table S12. The reacted antibodies were detected using a VECTASTAIN Elite ABC kit for rabbit or rat IgG (Vector Laboratories, Burlingame, CA, USA) according to the manufacturer's instructions. The staining of OPN, MCP-1, superoxide dismutase (SOD), APN were measured for 6 kidneys, and expressed as ratios (%) of the total tissue area of kidney cross-sections using Image-Pro Plus software (Medica Cybernetics Inc., Bethesda, MD, USA).

### Western blot analysis

Whole-protein extracts from specimens were immersed in 1× lysis buffer and lysed by sonication on ice. The lysate was cooled on ice for 15 min and then clarified by low-speed centrifugation (1,000× *g*). The total protein concentration in the supernatant was spectrophotometrically quantified using an Ultrospec 3100 pro (GE Healthcare, Wallingford, CT, USA). Samples containing 30 µg total protein were mixed with loading buffer (Laemmli Sample Buffer; Bio-Rad Laboratories, Hercules, CA, USA) and boiled for 10 min. Proteins were resolved by 12.5% sodium dodecyl sulfate-polyacrylamide gel electrophoresis (SDS-PAGE) and transferred onto Immobilon®-Polyvinylidene fluoride (PVDF) membranes (Millipore, Bedford, MA, USA). Non-specific binding on the membranes was blocked for 1 h at room temperature by using Tris-buffered saline (pH 7.5)-Tween 20 containing 5% skim milk, followed by an overnight incubation at 4°C with the antibodies listed in Table S12.

### TUNEL-positive cells counting

Images of sections were scanned and expressed as number of the total cortico-medulla junction of kidney cross-sections by using Image-Pro Plus software (Medica Cybernetics Inc., Bethesda, MD, USA). Cell counts were done by two researchers in a blinded fashion. To count cells, the slides were projected onto a grid comprising 12 fields. Six randomly chosen fields were used. These six fields were used for all study slide counts [18]. Magnification is ×400.

### Statistical analysis

The amount of kidney crystal deposition and immunohistochemical staining deposition and the results of serum and urine tests are shown as means ± SD. The values of mRNA expression of all genes, measured by quantitative RT-PCR, are shown as means ± SE. The statistical significance of differences between groups was examined using the Mann-Whitney U test, and a probability of 0.05 was taken as significant.

## Results

### Serum and urine biochemistry

At day 0, the total cholesterol (TC) values in ob/ob mice were significantly higher than those in +/+ mice (Table S1). None of the other determined values were significantly different between the 2 groups. At day 6, the triacylglyceride (TG) and TC levels in ob/ob mice were substantially higher than those in wild-type mice. Moreover, the TC and free fatty acid (FFA) values in ob/ob mice were significantly higher than those in wild-type mice. At day 0, the serum APN value in ob/ob mice was lower than that in wild-type mice. Moreover, APN was decreased by glyoxylate administration. The plasma APN levels after recombinant APN injection were similar to physiological levels (Table S1). APN treatment did not result in any significant changes in serum biochemistry results.

### Kidney crystal depositions

No crystal formation could be detected in +/+ kidneys at days 0 and 6. CaOx crystal depositions were detected in the renal proximal tubular lumen located at the region between the renal cortex and the medulla only in ob/ob kidneys at day 6 (Fig. 1A). APN treatment ameliorated crystal aggregation and scattered the crystals throughout the entire kidney region. A quantitative evaluation of kidney crystal formation at day 6 revealed the amount of the crystals in ob/ob kidneys was significantly higher than that in +/+ kidneys (p = 0.0004) and APN-treated ob/ob kidneys (p = 0.005) (Fig. 1B).

**Figure 1:** Detection and quantification of calcium oxalate kidney crystal formation. A. Kidney sections of wild type (+/+), obesity (ob/ob), and adiponectin-treated ob/ob (ob/ob+APN) mice at day 6. The upper images show calcium oxalate crystal deposits in Pizzolato-stained sections. The lower images show non-stained sections observed by polarized light optical microphotography (PLOM). Magnification is ×20 (in box: ×400). B. Quantification of kidney crystals in +/+, ob/ob, and ob/ob+APN mice. Data are indicated as the mean ± SD. a; p = 0.0004, b; p = 0.005.

### Microarray analysis and data mining

A genome-wide expression assay using microarrays indicated 45,101 genes were significantly changed in expression. Based on the schema of Fig. 2A, the number of gene groups with >2.0-fold increased and <0.5-fold decreased expression between the relevant groups was as follows: *ΔA* (gene expression involving GOx administration), 157 and 159 genes; *ΔB* (gene expression involving obesity), 186 and 218; *ΔC* (gene expression involving GOx administration and kidney crystal formation), 621 and 627; *ΔD* (gene expression involving obesity and kidney crystal formation), 662 and 817; *ΔE* (gene expression involving obesity, GOx administration, and kidney crystal formation), 668 and 895; and *ΔF* (gene expression involving APN administration and kidney crystal prevention), 190 and 154.

**Figure 2:** The scheme of the microarray analysis design. A. Experimental design and gene expression changes between groups. *Δ* refers to a gene group with >2.0- or <0.5-fold expression change between 2 experimental groups. *ΔA* means gene expression involving GOx administration. *ΔB* means gene expression involving obesity. *ΔC* means gene expression involving GOx administration and kidney stone formation. *ΔD* means gene expression involving obesity and kidney stone formation. *ΔE* means gene expression involving obesity, GOx administration, and kidney stone formation. *ΔF* means gene expression involving APN administration and kidney stone prevention. +GOx, glyoxylate administration; +APN, adiponectin treatment. B. The selection scheme for kidney stone formation-related gene groups (Venn diagram). The gray-stained area is represented by (*ΔC*∩*ΔD*∩*ΔE*)\(*ΔA*∪*ΔB*) and is the kidney stone formation-specific gene group under a MetS environment.

Among the genes with increased expression (Table S2) were inflammatory-related genes such as lipocalin 2 (*Lcn2*) and cell cycle-related genes such as minichromosome maintenance deficient 5 (*Mcm5*). Among the genes with decreased expression (Table S4) were those from the solute career family (Slc12a1, Slc7a13). GO analyses were performed for the genes showing increased and decreased expression during kidney crystal formation (Tables S3 and S5, respectively). The upregulated genes belonged to the categories related to inflammation and immunoresponse, collagen production, and cell proliferation with DNA replication. Meanwhile, the downregulated genes belonged to the categories related to oxidoreductase and oxygen transporter activity and to chromatin and nucleosome assembly.

Among the kidney crystal-related genes, those that showed a reversal in their expression through exogenous APN treatment were selected, i.e., the genes among the >2.0-fold upregulated genes related to kidney crystal formation that showed a <0.5-fold reduction in expression with APN treatment [((*ΔCi*∩*ΔDi*∩*ΔEi*)\(*ΔAi*∪*ΔBi*))∩*ΔFd*], and vice versa for the genes among the <0.5-fold downregulated genes related to kidney crystal formation [((*ΔCd*∩*ΔDd*∩*ΔEd*)\(*ΔAd*∪*ΔBd*))∩*Δfi*]. The number of genes belonging to each group was 154 and 190, and the top 10 genes with the highest and lowest expression changes between the ob/ob and ob/ob+APN groups at day 6 are listed in Tables S6 and S8. The downregulated genes belonged to the categories related to immunoreactions with T-cell proliferation via IL-11 binding (Table S7); the upregulated genes, to the categories related to mitosis and the cell cycle and to oxidoreductase and oxygen transporter activity (Table S9).

### Expression of kidney crystal-related genes (Spp1, Ccl2, Sod2) and Adipoq

The expression changes in *Spp1*, *Ccl2*, and *Sod2*, previously reported as kidney crystal formation-related genes, and *Adipoq* were evaluated by quantitative PCR (Fig. 3A). The expression of the encoded proteins (OPN, MCP-1, SOD, and APN, respectively) was subsequently examined using immunohistochemistry (Fig. 3B).

**Figure 3:** Expression analyses of *Spp1*, *Sod2*, *Ccl2*, and *Adipoq*. A. The results of quantitative PCR for the expression of *Spp1*, *Sod2*, *Ccl2*, and *Adipoq*. Expression levels are expressed relative to *Actb* (*actin-beta*) transcript levels. *Spp1*, secreted phosphoprotein 1; *Ccl2*, C-c chemokine ligands 2; *Sod2*, superoxide dismutase 2; *Adipoq*, adiponectin. Data are indicated as the mean ± SE. *, p<0.05 between groups at the same time point. †, p<0.01 compared with the same group at day 0. B. Immunohistochemical staining for OPN, MCP-1, SOD, and APN expression. OPN, osteopontin; MCP-1, monocyte chemotactic protein-1; SOD, superoxide dismutase; APN, adiponectin. Magnification is ×20 (in box: ×400). C. The quantification of immunohistochemical staining. Data are indicated as the mean ± SD. *, p<0.05 between groups at the same time point. †, p<0.05 compared with the same group at day 0.

*Spp1* in ob/ob mice displayed relatively higher expression than in +/+ mice at day 0. This difference became significant at day 6 (2.60-fold, p = 0.020). *Spp1* expression in +/+ mice showed a relative increase after GOx administration (2.10-fold, p = 0.070). Meanwhile, *Spp1* in ob/ob mice increased significantly with kidney crystal formation (1.91-fold, p = 0.030), and the expression value did not change following exogenous APN treatment. *Ccl2* expression demonstrated no significant difference between ob/ob and +/+ mice at day 0. However, its expression in ob/ob mice increased significantly at day 6 (14.59-fold, p = 0.004) compared to day 0 but showed no remarkable change in +/+ mice. APN treatment did not change *Ccl2* expression values in ob/ob mice. *Sod2* expression at day 0 showed no significant difference between both genotypes; however, its expression in ob/ob mice decreased significantly at day 6 (0.31-fold, p = 0.008). Further, the decreased *Sod2* expression could not be recovered by exogenous APN treatment. The expression of *Adipoq* in ob/ob mice at day 0 was significantly lower than that of +/+ mice (0.17-fold, p = 0.046), and the expression in +/+ mice was significantly decreased by GOx administration at 6 days (without crystal formation) (0.25-fold, p = 0.049).

The expression of stone related protein and endogenous APN demonstrated by immmunohistochemistry (Fig. 3B) followed the result of quantitative PCR. OPN was focally present at the renal cortical proximal tubular cells for both genotypes at day 0. Its expression expanded in a somewhat diffuse manner and centered around the cortico-medullar border region at day 6, especially in the ob/ob and ob/ob+APN groups with crystal formation. MCP-1 expression was clearly detected, especially in the cortical proximal tubular cells at day 0, and its expression in ob/ob mice showed a remarkable increase at the cortico-medullar border regions. MCP-1 expression in the ob/ob+APN group showed a similar distribution but appeared to be weaker than that of the ob/ob group. For both genotypes, SOD was expressed in the proximal tubular cells at the cortico-medullar junction area at day 0. Its expression intensity at day 6 was almost unchanged in the +/+ group but decreased remarkably in the ob/ob and ob/ob+APN groups. At day 0, endogenous APN in the +/+ mice could be detected strongly in the interstitial cells at the renal papilla and also in the renal parenchyma. However, the ob/ob mice at day 0 showed a remarkably lower number of APN-positive interstitial cells than +/+ mice. All groups at day 6 showed a reduced number of APN-positive interstitial cells. The results of the quanitification of immunohistochemical staining were similar to the expression of stone related genes and APN.

### Confirmation of the selected genes detected by microarray analysis

Among the selected genes with significant expression changes in the microarray analysis, the expression of several characteristic genes belonging to 5 or 6 categories based on GO analysis was evaluated by quantitative PCR (Fig. 4A–E), identified several genes that were affected by APN treatment, and they were evaluated by immunohistochemistry (Fig. 5A–F). and western blotting (Fig. 6)

**Figure 4:** Confirmation that selected genes detected by microarray analysis showed differential expression between different treatment groups. The expression of several characteristic genes belonging to 5 categories based on GO analysis was evaluated by quantitative PCR. Expression levels are expressed relative to *Actb*. Data are indicated as the mean ± SE. *, p<0.05 between the groups at the same time point. †, p<0.01 compared with the same group at day 0. 5 categories are as follows. A. Inflammation and immune-related gene group: *Lcn2*, lipocalin2; *Cd44*, CD44 antigen; *Lyz1*, lysozyme1. B. Apoptosis-related gene group: *Stat3*, signal transducer and activator of transcription 3; *Aurka*, aurora kinase A. C. Cell repair and proliferation-related gene group: *Mcm5*, minichromosome maintenance deficient 5. D. Adhesion and fibrosis-related gene group: *Vcam1*, vascular cell adhesion molecule 1; *Col3a1*, collagen, type III, alpha 1. E. Transporter-related gene group: *Slc12a1*, solute carrier family 12, member 1; *Slc7a13*, solute carrier family 7, member 13.

**Figure 5:** Confirmation of selected genes detected by microarray analysis. A–F. Among the selected genes with significant expression changes in the microarray analysis, the expression of several characteristic genes belonging to 6 categories based on GO analysis was evaluated by immunohistochemical staining. Magnification is ×20 (in box: ×400). 6 categories are as follows. A. Inflammation and immune-related gene group: LYZ1, Lysozyme 1.CD44, CD44 antigen; MHC-class 2, major histocompatibility complex-class2. B. Apoptosis-related gene group: STAT3, signal transducer and activator of transcription 3; AURKA, aurora kinase A, Thymidine kinase 1, C. Cell repair and proliferation-related gene group: MCM5, minichromosome maintenance deficient 5. D. Adhesion and fibrosis-related gene group: Fn, Fibronectin. E. Oxidative stress-related gene group: 8OHdG, 8-Hydroxydeoxyguanosine. F: transporter-related gene group; SLC12A1, solute carrier family 12, member 1.

**Figure 6:** Confirmation of selected genes detected by microarray analysis. Western blot analysis for OPN, MCP-1, SOD, APN, LYZ1, AURKA, TK1, MCM5, NGAL, CD44, STAT3, SLC12A1, SLC7A13, VCAM1, COL3A1 and FN protein expression. Each molecular weight demonstrated as the bands were as follows. OPN, 75 and 55 kDa; MCP-1,17 kDa; SOD, 37 kDa; APN, 64 kDa; LYZ1, 17 kDa; AURKA, 40 kDa; TK1, 25 kDa; MCM5, 90 kDa; NGAL, 25 kDa; CD44, 80–95 kDa; STAT3, 92 kDa; SLC12A1, 47 kDa; SLC7A13, 52 kDa; VCAM1, 100 kDa; COL3A1, 138 kDa; FN, 212 kDa and β-actin, 37 kDa.

GOx administration resulted in the significant upregulation of *Lcn2*, *Cd44*, and *Lyz1* in ob/ob and +/+ mice at day 6. For *Cd44* and *Lyz1*, kidney crystal formation further enhanced their expression, as their transcript levels were significantly higher in ob/ob mice than in +/+ mice. APN treatment resulted in a relative decrease in *Lcn2* and *Cd44* expression and a significant decrease in *Lyz1* expression in ob/ob mice (Fig. 4A).

*Stat3* expression in ob/ob mice was significantly higher at day 6 than day 0 (Fig. 4B). APN treatment did not induce a remarkable change in *Stat3* (Fig. 4B). *Aurka* significantly increased at day 6 in both genotypes and significantly increased with exogenous APN treatment. In ob/ob mice, *Tk1* expression showed significant higher expression at day 6 relative to day 0 and significantly increased with exogenous APN treatment.

Meanwhile, *Mcm5* expression significantly increased at day 6 in both genotypes and significantly increased with exogenous APN treatment (Fig. 4C).

Following GOx treatment, *Vcam1* and *Col3a1* were significantly upregulated. Kidney crystal formation further enhanced *Vcam1* expression in ob/ob mice at day 6 when compared to wild-type mice. APN treatment resulted in relatively decreased *Vcam1* and *Col3a1* expression (Fig. 4D).

*Slc12a1* and *Slc7a13* were significantly downregulated in the presence of kidney crystal formation in ob/ob mice at day 6, showing significantly reduced levels compared to wild-type mice (Fig. 4E). Moreover, APN treatment did not induce a remarkable change in the expression of *Slc12a1* and *Slc7a13* (Fig. 4E).

Fig. 5A shows inflammation and immune-related protein expression for NGAL, CD44, LYZ1, F4/80, mouse macrophage surface marker, and major histocompatibility complex-class 2 (MHC-class 2). NGAL was barely detectable at day 0 and was observed in the proximal tubular cells from the cortex to the papilla. LYZ1 and CD44 were detected at the interstitium and at the proximal tubular cells from the cortex to the papilla in a diffuse manner at day 0. At day 6, these expressions strengthened focally at the cortico-medullary junction where kidney crystals were formed. This tendency was also particularly enhanced in ob/ob and ob/ob+APN mice. F4/80 was barely detectable at day 0 and was observed in interstitial cells from the cortex to the papilla. In ob/ob mice at day 6, MHC-class 2 showed particularly strong expression around the cortico-medulla junction area. MHC-class 2 expression indicates macrophage activity. MHC-class 2 could not be detected at day 0. However, it localized to interstitial and proximal tubular cells at cortico-medullary junction and in ob/ob kidneys at day 6. MHC-class 2 expression levels were lower in ob/ob+APN kidneys than in ob/ob ones at day 6.

Fig. 5B shows apoptosis-related protein expression for signal transducer and activator of transcription 3 (STAT3), aurora kinase A (AURKA), Thymidine kinase 1 (TK1), as well as TUNEL staining as an apoptosis index. STAT3 at day 0 was present in a diffuse manner in renal proximal tubular cells from the cortex to the medulla for both genotypes. In ob/ob kidneys at day 6, focal staining at the crystal formation area of the cortico-medullary junction was observed. At day 6, the expression in ob/ob+APN kidneys compared to ob/ob ones. AURKA expression was detected in the proximal tubular cells at the area of the cortex-medulla, and ob/ob and ob/ob+APN kidneys at day 6 showed strong expression at the cortico-medullary junction area. TK1 at day 0 was present in a diffuse manner in renal proximal tubular cells from the cortex to the medulla for both genotypes. In ob/ob kidneys at day 6, focal staining at the crystal formation area of the cortico-medullary junction was observed. At day 6, the expression in ob/ob+APN kidneys compared to ob/ob ones.

MCM5 was hardly detected at day 0 but showed strong expression in the nuclei of proximal tubular cells in the area from the cortex to the papilla at day 6, particularly in ob/ob+APN kidneys (Fig. 5C).

Fig. 5D shows the expression of the adhesion and fibrosis-related protein fibronectin (Fn) as a fibrosis index. Fn expression showed a diffuse localization pattern in the interstitial cells from the cortex to the papilla. At day 6, both ob/ob and ob/ob+APN kidneys showed strong expression around the crystal-forming area, with the latter showing relatively weaker expression than the former.

Fig. 5E shows an oxidative stress-related index for 8-hydroxydeoxyguanosine (8-OHdG). 8OHdG was detected in the nuclei of the proximal tubular cells in the area from the cortex to the papilla, with ob/ob and ob/ob+APN kidneys at day 6 showing strong expression. The former showed weaker staining than the latter.

Transporter-related solute career family 12, member 1 (SLC12A1) was expressed diffusely through the entire kidney in both genotypes at day 0 (Fig. 5F). At day 6, ob/ob and ob/ob+APN kidneys showed diminished expression at the cortico-medullary junction area where kidney crystals were formed.

By TUNEL staining, ob/ob and ob/ob+APN kidneys at day 6 showed stained nuclei in the area from the cortex to medulla, with the cortico-medullary junction showing particularly strong staining. At day 6, ob/ob+APN kidneys showed weak staining compared to ob/ob ones. At day6, TUNEL-positive cells increased significantly in ob/ob mice. In ob/ob+ APN mice, the number of TUNEL-positive cells was lower than that in ob/ob mice (Fig. 7).

**Figure 7:** TUNEL staining and the number of TUNEL-positive cells. Data are indicated as the mean ± SD. *, p<0.05 between groups at the same time. **, p<0.01 between groups at the same time point. †, p<0.01 compared with the same group at day 6.

The results of western blot analysis were similar to immunohistochemical staining in OPN, MCP-1, SOD, APN, LYZ1, AURKA, STAT3, MCM5 and SLC12A1 and were similar to the expression in OPN, MCP-1, SOD, APN, LYZ1, AURKA, TK1, MCM5 and SLC12A1.(Fig. 6). All of our findings by RT-PCR, immunohistochemical staining and western blotting were summalized in Table S10.

## Discussion

In the present study, we investigated the following 3 points to elucidate the mechanism of kidney crystal formation under the MetS environment as well as the efficacy of exogenous APN treatment as an MetS prophylactic agent for kidney crystal prevention: (i) mineral environmental changes in blood and urine, (ii) expression changes and renal distribution of previously reported kidney crystal-related genes and endogenous APN, and (iii) novel genetic environmental changes in the kidney by using a genome-wide analysis.

Serum and urine biochemistry data indicated a high concentration of serum TC and triglyceride TG in MetS model mouse (ob/ob mouse). However, as previously reported, a decrease in urinary pH or citrate [19] or an increase in urinary calcium, uric acid, or oxalate concentration was not observed [20].

Next, changes in the expression of previously reported kidney crystal-related genes were investigated. Before kidney crystal formation, the kidneys in ob/ob mice showed significantly higher expression of OPN and significantly lower expression of endogenous APN than kidneys from +/+ mice. At day 6, the +/+ kidneys without crystals showed a slight increase in OPN expression and a decrease in SOD expression, but the expression of MCP-1 did not change remarkably. However, the expression of endogenous APN in the +/+ mice significantly decreased. This change might be the result of factors involved in the mechanism linking GOx administration with crystal formation. The lower value for endogenous APN expression at day 0 probably caused kidney crystal formation in ob/ob mice. Thus, the suppression of APN expression resulted in the progression of kidney crystal formation. In this study, we found that APN expression was localized in the renal interstitial cells, which possess lipid drops that produce prostaglandins and prostacyclins in the cytoplasm [21]. It is reported that APN is mainly produced from the adipose tissue [22]. We observed APN expression was decreased in ob/ob mouse and the kidney crystal formation kidneys in this study, but it is unclear whether the kidney-specific APN was more important for kidney crystal formation than adipocytes-derived one. The details regarding the physiological functions of the cells remain unclear.

Previous studies indicate that hypertrophy of adipocytes decreased exogenous APN expression. Tsuchida *et al.* [23] reported that the control of APN receptor sensitivities via the Insulin/Foxo1 pathway might be involved in the progression of oxidation and inflammation via deficiency of APN. Recently, Shibata *et al.* [24] reported a protective effect for APN in mitochondrial injury of cardiac myocytes. In the present study, we showed that exogenous APN treatment could prevent kidney crystal formation. However, APN treatment could not induce significant changes in the expression of “traditional” crystal-related genes such as *Spp1*, *Ccl2*, and *Sod2*. These results indicate that the crystal-preventive effect of APN treatment did not involve suppression of SOD-related oxidative stress, MCP-1-related inflammation, or OPN-related crystal matrix expression. Commonly, inflammation suppressed APN excretion from adipocytes via macrophage-derived Il-6 and TNF-alpha expression. Our previous study showed that kidney crystal formation was accompanied by inflammation involving OPN and MCP-1 expression, and induced macrophage migration to renal interstitium [25]. Our genome-wide study using stone model mice indicated increased expression of Il-6 and TNF-alpha during kidney crystal formation [26]. This might be the reason of decreased APN expression during kidney crystal formation.

In the microarray analysis, among the extracted functional categories by GO analysis, inflammation and immune-related genes were noticeable. Among the inflammation-related genes, *Lyz1* showed significantly decreased expression following APN treatment. *Lyz1*, which was also detected by our previous genome-wide analysis using a crystal formation mouse model, is a macrophage-derived hydrolase and a component of the crystal matrix [26].

Based on the results of the TUNEL staining, APN treatment may improve apoptosis; however, STAT3 expression did not change with APN treatment. In contrast, AURKA, an antiapoptotic agent in the p73-dependent apoptosis pathway [27], was upregulated significantly at day 6, while the expression of this protein in ob/ob kidneys was significant lower than that in +/+ kidneys. Hence, the MetS environment may suppress the antiapoptosis ability of Aurka, and APN treatment may significantly recover its expression. Thymidine kinase 1 (TK1) is a cytoplasmic enzyme functioning in phosphorylation and DNA synthesis and acts in renoprotection against apoptosis [28]. In this study, TK1 might play important roles in the repair of injured proximal tubular cells by GOx, and APN treatment may improve this ability, leading to renoprotection against crystal formation.

For examining cell repair and proliferation, we investigated MCM5 expression during kidney crystal formation. As suggested by this study, MCM5 might play important roles in repairing proximal tubular cells injured following GOx, and APN treatment may improve this ability, leading to renoprotection from crystal formation.

We investigated the production of 8-OHdG as an index of oxidative stress, 8-OHdG is one of the major forms of DNA damage induced by reactive oxygen species [29]. The pattern of 8-OHdG production was similar to *Sod2* expression, and APN was unable to inhibit the oxidative stress.

On the basis of these research findings, the decrease of serum and renal APN was thought to be one of the factors in process of crystallization. However, only by a decrease of APN, we think another formation mechanism under MetS.

## Conclusions

This study provided compelling evidence indicating that the mechanism of kidney crystal formation in the MetS environment involved renal biomolecular environmental changes, including increased expression of inflammation molecules such as OPN, and decreased transporter activities due to accumulated oxidative stress and cell injury. The genome-wide analysis suggests that the mechanism of kidney crystal formation in the MetS environment does not involve changes in urinary mineral composition. Moreover, we showed that exogenous APN treatment significantly prevented kidney crystal formation and that the mechanism involved renoprotective functions via anti-inflammatory and antiapoptotic effects and injured cell repair functions. Therefore, APN might be an effective prophylaxis not only for atherosclerosis but also for kidney crystal formation.

## Supporting Information

Table S1 **Serum and urine biochemistry.** Serum and urine biochemistry in +/+ and ob/ob mice (n = 6) on days 0 and 6. Each value is the mean ± SD value, n = 6. *p<0.05 versus +/+ on day 0. **p<0.01 versus +/+ on day 0. †*p*<0.05 versus +/+ on day 6.
(TIF)

Table S2 **Ten genes showing the greatest increase in expression in the kidney stone formation-related gene group.** Listed genes showed a >2-fold change. Fold change compared with the controlled raw value of +/+ mice on day 0. Gray-toned genes are followed by quantitative PCR or immunohistochemistry.
(TIF)

Table S3 **GO analysis of overexpressed genes in the kidney stone formation-related gene group.** The 259 genes were clustered based on their GO biological process, cellular component, and molecular function ontology. Within the top 10 of each category, the GO with the lowest p-value was selected.
(TIF)

Table S4 **Ten genes with the greatest decrease in expression in the kidney stone formation-related gene group.** Listed genes showed a <0.5-fold change. Fold change compared with the controlled raw value of +/+ mice on day 0. Gray-toned genes are followed by quantitative PCR or immunohistochemistry.
(TIF)

Table S5 **GO analysis of genes with suppressed expression in the kidney stone formation-related gene group.** The 243 genes were clustered based on their GO biological process, cellular component, and molecular function ontology. Within the top 10 of each category, the GO with the lowest p-value was selected.
(TIF)

Table S6 **Twelve genes with the greatest expression decrease in the >2.0-fold upregulated genes related to kidney stone formation and the <0.5-fold downregulated gene group by APN treatment.** Fold change compared with the controlled raw value of ob/ob mice on day 6. Gray-toned genes are followed by quantitative PCR or immunohistochemistry.
(TIF)

Table S7 **GO analysis of genes with suppressed expression in the >2.0-fold upregulated genes related to kidney stone formation, <0.5x downregulated gene group by APN treatment.** The 154 genes were clustered based on their GO biological process, cellular component, and molecular function ontology. Within the top 10 of each category, the GO with the lowest p-value was selected.
(TIF)

Table S8 **Ten genes from the <0.5-fold downregulated genes related to kidney stone formation, with the highest expression increase on APN treatment, >2.0-fold upregulated gene group.** Fold change compared with the controlled raw value of ob/ob mice on day 6. Gray-toned genes are followed by quantitative PCR or immunohistochemistry.
(TIF)

Table S9 **GO analysis of genes from the <0.5-fold downregulated genes related to kidney stone formation that were overexpressed on APN treatment, >2.0-fold upregulated gene group.** The 190 genes were clustered based on their GO biological process, cellular component, and molecular function ontology. Within the top 10 of each category, the GO with the lowest p-value was selected.
(TIF)

Table S10 **The expression changes of genes and proteins by GOx administration, obesity, and APN administration. ↑↑; more increased, ↑; increased, →; no remarkable change, ↓; decreased, ↓↓; more decreased.** Gray-toned genes are followed significantly changes by APN administration.
(TIF)

Table S11 **Gene title, Protein name and Taqman MG probe ID TaqMan Gene Expression Assay (Applied Biosystems, Foster City, CA,USA), 20× assay mix of primers, and TaqMan MG probes (FAM dye labeled; Applied Biosystems) were used for quantitative RT-PCR.** This assay was designed to span exon–exon junctions so as not to detect genomic DNA. Validation experiments were performed to test the efficiency of the target amplification and reference amplification.
(TIF)

Table S12 **The antibodies' name.**
(TIF)
